The article "C-Reactive Protein as a Prognostic Biomarker for Gynecologic Cancers: A Meta-Analysis" was retracted in 2023. Reasons: signs of a paper mill; suspected computer-generated content; unreliable results or conclusions; concerns about the data.

# C-Reactive Protein as a Prognostic Biomarker for Gynecologic Cancers: A Meta-Analysis

**DOI:** 10.1155/2022/6833078

**Published:** 2022-10-11

**Authors:** Yingying Yang, Xiu Li, Hui Qian, Guangci Di, Ruhua Zhou, Yuwei Dong, Wenyue Chen, Qingling Ren

**Affiliations:** ^1^Department of Gynaecology, Affliated Hospital of Nanjing University of Chinese Medicine, No. 155, Hanzhong Street, Nanjing 210029, Jiangsu, China; ^2^Department of Gastroenterology, Affliated Hospital of Nanjing University of Chinese Medicine, No. 155, Hanzhong Street, Nanjing 210029, Jiangsu, China; ^3^Nursing Institute of Nanjing Medical University, No. 818, Tianyuan Street, Nanjing 210029, Jiangsu, China

## Abstract

**Background:**

The prognostic role of CRP (C-reactive protein) in gynecological tumors has been previously reported in individual studies, but whether CRP can be used as a separate potential prognostic factor has not been systematically reviewed. The purpose of this research is to determine if there is a link between CRP levels and the prognosis of gynecological cancer patients.

**Methods:**

A systematic search was carried out to find the literature evaluating the predictive role of CRP in the prognosis of gynecological cancer patients. For the purpose of determining the relationship between CRP and clinicopathological characteristics, the pooled odds ratio (OR) was calculated. A hazard ratio (HR) with a 95% confidence interval (CI) was used to determine differences in overall survival (OS), disease-free survival (DFS), or progression-free survival (PFS) between patients with low and high CRP levels.

**Results:**

A total of 19 studies, including 4062 patients, were analyzed retrospectively. The FIGO stage was related to the CRP level (OR = 0.43, 95% CI: 0.19–1.00). Age, lymph node metastasis, and histological grade were not associated with CRP level (OR = 0.93, 95% CI: 0.69–1.25; OR = 0.91, 95% CI: 0.65–1.28; OR = 0.74, 95% CI: 0.52–1.05). Worse OS (HR = 1.40, 95% CI: 1.23–1.57), DFS (HR = 1.20, 95% CI: 1.12–1.28), and PFS (HR = 1.57, 95%CI: 1.23–1.91) were associated with elevated CRP levels, as shown by the pooled results. Subgroup analysis was performed according to cancer type (endometrial cancer: HR = 1.15, 95% CI: 1.02–1.28; ovarian cancer: HR = 1.67, 95% CI: 1.03–2.31; cervical cancer: HR = 1.42, 95% CI: 1.19–1.64), multivariate value (HR = 1.22, 95% CI: 1.10–1.33), and age (HR = 1.50, 95% CI: 1.28–1.72). Significant correlations were observed between CRP and OS.

**Conclusions:**

CRP may be utilized as a prognostic indicator for a variety of gynecologic malignancies, including cervical cancer, ovarian cancer, endometrial cancer, and vulvar cancer.

The article "C-Reactive Protein as a Prognostic Biomarker for Gynecologic Cancers: A Meta-Analysis" was retracted in 2023. Reasons: signs of a paper mill; suspected computer-generated content; unreliable results or conclusions; concerns about the data.

## 1. Introduction

In 2020, there have been more than 135000 verified instances of three main gynecological malignancies worldwide. These include cervical cancer, ovarian cancer, and endometrial cancer. The fourth most common cause of cancer-related mortality in women is cervical cancer. [1]. Chinese and Indian cases account for one-third of the total in the world [2]. The incidence and mortality of cervical cancer will decrease due to the extensive implementation of the cytology screening programs. Ovarian cancer is the seventh most frequent female cancer in the world, according to the World Health Organization. In 2020, there emerged 310000 new cases of ovarian cancer and 210000 deaths worldwide. Ovarian cancer has a morbidity of 1/75 and mortality of 1/100 [3]. Ovarian cancer is usually diagnosed at its advanced stage, which leads to high mortality. The five-year relative survival rate is barely 29%. Approximately 15% of cases are identified as localized cancers (stage 1), with a 5-year survival rate of 92%. Globally, the 5-year relative survival rate is between 30% and 40%, with just a little improvement (2–4%) since 1995 [4]. In 2021, 420,000 new cases of endometrial cancer were reported worldwide [5]. The incidence and mortality of endometrial cancer have been progressively rising in most developed nations, mostly as a result of changes in lifestyle, the aging population, and socioeconomic factors. Gynecological cancers are mainly treated with surgery, radiotherapy, chemotherapy, biological, and targeted drugs. Postoperative markers, which include histopathological grade, lymph node status, and invasion depth, are viewed as vital indicators of the progression and recurrence of gynecological cancers [6]. However, radiotherapy and chemotherapy pose a high toxic burden and an economic cost. Therefore, more biomarkers should be explored to reform the current treatment strategies.

The role of chronic inflammation in carcinogenesis has been widely studied. The relationship between inflammation and tumorigenesis was first proposed by Rudolph Virchow in 1863 [7]. Furthermore, several inflammatory indicators, such as C-reactive protein (CRP), have been shown to be able to predict the prognosis of some cancers, including gastric cancer and lung cancer [8]. Recent research has confirmed that serum CRP levels are positively related to the degree of malignancy [9–18].

CRP is a protein that is produced by hepatocytes during the acute phase of an inflammatory response. Its level rises sharply to remove pathogens and activate the complement system. Many malignant tumors occur in chronically infected tissues, and 15–20% of human tumors are related to inflammation [12]. Patients with malignant tumors may have a rise in serum CRP levels, which may be associated with the proliferation of tumor cells and the generation of inflammatory substances in the body. Some proinflammatory cytokines, such as IL-6 and IL-11, can stimulate the expression of CRP, resulting in an increase in serum CRP levels [13–16].

The article "C-Reactive Protein as a Prognostic Biomarker for Gynecologic Cancers: A Meta-Analysis" was retracted in 2023. Reasons: signs of a paper mill; suspected computer-generated content; unreliable results or conclusions; concerns about the data.

Higher CRP levels have been shown to be associated with a worse prognosis in a range of malignant tumors, including lung cancer, gastric cancer, and hepatic cancer. [17, 18]. However, its prognostic value in gynecological cancer is not clear. Therefore, the goal of this meta-analysis was to determine whether or not CRP affects a patient's prognosis after being diagnosed with gynecology cancer.

## 2. Materials and Methods

### 2.1. Data Collection

PubMed, Web of Science, and Embase were used to search for studies on CRP and gynecological cancer published before June 1, 2022. The following key words were used for literature retrieval: (“CRP” or “C-reactive protein”) and (“gynecologic” or “cervix uteri” or “corpus uteri” or “ovary” or “endometrium” or “vagina” or “vulva” or “fallopian tube” or “gynecological” or “cervical” or “ovarian” or “endometrial” or “vulvar” or “vaginal” or “GTD”), and (“tumor” or “carcinoma” or “cancer”). Additionally, the references in the obtained papers were scrutinized to find any other relevant research outside of these two key phrases in the query. The literature retrieval flowchart is shown in Figure 1.

### 2.2. Inclusion Criteria

Inclusion criteria were those studies in which (a) the postoperative pathological diagnosis of gynecologic cancer was made; (b) the serum CRP prior to and/or after the surgery was assessed; (c) serum CRP was measured; (d) clinical-pathological characteristics, prognosis, stage, or grade of gynecologic cancer were studied in connection to CRP expression in the serum.

Exclusion criteria were those studies in which (a) useful data could not be extracted; (b) the survival data or 95% confidence interval (CI) was not reported; (c) only editorials, reviews, and comments were available. In addition, when the data of a patient were used in multiple studies, we select the latest study.

### 2.3. Extraction of Data and Evaluation of Quality

The data from the eligible studies were carefully examined by independent researchers YY. Y, RH. Z, H. Q and X. L. The data extracted mainly included: the first author, publication date, sample size, the cancer type, country, recurrence, average age, duration of follow-up, tumor pathologies, FIGO stage, cut-off value for CRP, and outcomes of patients (overall survival (OS), disease-free survival (DFS), recurrence-free survival (RFS), progress-free survival (PFS)), and disease-specific survival (DSS)). The Newcastle-Ottawa Scale was also utilized to assess the overall quality of the publications' included articles.

The article "C-Reactive Protein as a Prognostic Biomarker for Gynecologic Cancers: A Meta-Analysis" was retracted in 2023. Reasons: signs of a paper mill; suspected computer-generated content; unreliable results or conclusions; concerns about the data.

### 2.4. Statistical Analysis

The statistical analysis was carried out with the help of Stata 12.0 (StataCorp LP). The OR and 95% CI were used to assess the correlations between serum CRP and clinicopathological characteristics. To further understand the predictive significance of CRP, we used pooled HRs with 95% CI intervals to analyze the relationship between CRP and survival. Multivariate analysis was preferred based on results from univariate analysis. If not reported directly in the literature, the HR with 95% CI was extrapolated from the Kaplan–Meier curves. *χ*^2^ and *I*^2^ tests were used to assess the heterogeneity across the articles. *p* < 0.10 or I2 > 50% indicated significant heterogeneity between studies, and these studies were deemed to be the best for building a random-effects model, rather than a fixed-effects model, for estimating the pooled ORs/HRs. In addition, a one-way sensitivity analysis was carried out to determine the stability of the current findings. The Begg test and funnel plots were also used to determine whether or not there was a difference in publication bias across the publications included. Among these two-tailed statistical tests, *p* < 0.05 (95% CI) was regarded as statistically significant.

## 3. Results

### 3.1. Characteristics of Included Studies

A total of 19 eligible studies were included, involving 4062 patients (1230 patients diagnosed with cervical cancer (CC), 1546 with ovarian cancer (OC), 1219 with endometrial cancer (EC), and 67 with vulvar cancer (VC)) [19–36]. It should be noted that all patients included in these studies received surgical treatment. Their basic characteristics are shown in Tables 1 and 2. The patients were from various countries, including Austria [19, 23, 28, 33, 36], China [20, 22, 24–26, 29, 31, 32, 34], Poland [21, 27], Japan [30, 35], and the United Kingdom [37]. These studies were published between 2007 and 2021 and their sample sizes could be traced. Various treatments, like surgery, radiotherapy, chemotherapy, and chemoradiotherapy, were used. In the articles above, the cut-off values of CRP ranged from 3.135 to 10 mg/L. In addition, OS, DFS, DSS, PFS, and RFS were described in 15, 4, 2, 3, and 2 studies, respectively.

### 3.2. Clinicopathological Characteristics and CRP

FIGO stage (OR = 0.43, 95% CI: 0.19–1.00; Table 3) (Figure 2(a)) was related to elevated CRP level. Age (OR = 0.93, 95% CI: 0.69–1.25; Table 3), histological grade (OR = 0.74, 95% CI: 0.52–1.05; Table 3), and lymph node metastasis (OR = 0.91, 95% CI: 0.65–1.28; Table 3) were not associated with elevated CRP level.

The article "C-Reactive Protein as a Prognostic Biomarker for Gynecologic Cancers: A Meta-Analysis" was retracted in 2023. Reasons: signs of a paper mill; suspected computer-generated content; unreliable results or conclusions; concerns about the data.

### 3.3. Long-Term Outcomes and CRP

High CRP levels were associated with worse OS (HR = 1.40, 95% CI: 1.23–1.57; *I*^2^ = 79.5%, *p* ≤ 0.001; Figure 2(b)), DFS (HR = 1.20, 95% CI: 1.12–1.28; *I*^2^ = 0.0%, *p* = 0.719; Figure 2(c)) and PFS (HR = 1.57, 95% CI: 1.30–1.98; *I*^2^ = 0.0%, *p* = 0.587; Figure 2(d)).

The subgroup analysis was based on groups that were stratified depending on the kind of cancer. There were statistically significant variations in the connection between CRP and OS of CC. (HR = 1.42, 95% CI: 1.19–1.64, *I*^2^ = 25.1%, *p* = 0.229; Figure 3(a)), OC (HR = 1.67, 95% CI: 1.03–2.31, *I*^2^ = 88.7%, *p* ≤ 0.001; Figure 3(a)) and EC (HR = 1.15, 95% CI: 1.02–1.28, *I*^2^ = 13.7%, *p* = 0.314; Figure 3(a)). A further subgroup analysis based on the HR value found that, when HR was treated as a multivariate variable, a moderately significant connection was detected between CRP and OS (HR = 1.22, 95% CI: 1.10–1.33, *I*^2^ = 26.7%, *p* = 0.235; Figure 3(b)). A subgroup analysis also confirmed significant correlation of OS with preoperative (HR = 1.50, 95% CI: 1.23–1.77, *I*^2^ = 74.6%, *p* ≤ 0.001; Figure 3(c)) and postoperative (HR = 1.31, 95% CI: 1.04–1.57, *I*^2^ = 68.9%, *p* = 0.004; Figure 3(c)) CRP. In the country-based subgroup analysis, significant correlations were observed between CRP and OS in western countries (HR = 1.39, 95% CI: 1.17–1.62, *I*^2^ = 76.3%, *p* ≤ 0.001; Figure 3(d)) or eastern countries (HR = 1.57, 95% CI: 1.18–1.96, *I*^2^ = 66.2%, *p* = 0.003; Figure 3(d)). In the age-based subgroup analysis, a significant correlation between CRP and OS was found among older patients (≥55 years old) (HR = 1.84, 95% CI: 1.30–2.38, *I*^2^ = 74.8%, *p* ≤ 0.001; Figure 3(e)), or younger patients (<55 years old) (HR = 1.31, 95% CI: 1.09–1.53, *I*^2^ = 70.1%, *p* ≤ 0.001; Figure 3(e)). In the CRP-based subgroup analysis, the correlation between CRP and OS was statistically significant (≤5 mg/L : HR = 1.28, 95% CI: 1.07–1.49, *I*^2^ = 58.5%, *p* = 0.047; Figure 3(f)), >5 mg/L : HR = 1.75, 95% CI: 1.24–2.26, *I*^2^ = 82.5%, *p* ≤ 0.001; Figure 3(f)).

### 3.4. Publication Bias and Sensitivity Analysis

Using the pooled data, a sensitivity analysis was performed in order to determine the relative contribution of each study to the estimated outcomes from that data (Figure 4). We found that the heterogeneity was not significant among the included studies. There was no evidence of publication bias, suggesting that the findings of the meta-analysis were statistically credible.

## 4. Discussion

CRP is mainly synthesized by the liver under the action of some proinflammatory factors [38]. It plays an important role in innate immunity, complement activation, and immunoglobulin receptor binding. The close correlation between CRP and the occurrence of malignant tumors has been widely recognized.

The article "C-Reactive Protein as a Prognostic Biomarker for Gynecologic Cancers: A Meta-Analysis" was retracted in 2023. Reasons: signs of a paper mill; suspected computer-generated content; unreliable results or conclusions; concerns about the data.

A meta-analysis has shown that mortality increases in patients with high CRP levels, particularly those with gastrointestinal malignancies and renal malignancies [39]. On the one hand, chronic inflammation can increase the risk of cancer. On the other hand, proinflammatory mediators and factors are released in cancer patients undergoing nonspecific inflammatory responses [40]. These mediators and factors can promote tumor growth and metastasis. At the same time, nonspecific inflammatory mediators caused by tumor tissue necrosis or (and) local tissue damage can regulate and induce hepatocytes to synthesize a large amount of CRP, resulting in a secondary increase in serum CRP concentration. The concentration of CRP not only reflects the degree of inflammatory response but also the malignancy of tumor phenotype and the possibility of metastasis [41]. According to the findings of this research, a rise in serum CRP levels is strongly associated with a higher FIGO stage, which is a significant prognostic factor.

IL-6 is produced by inflammatory processes, including cancer, and then, acts on the liver which produces C-reactive protein [42]. Based on these findings, it seems that serum CRP is a good alternative measure of IL-6 activity in cancer patients. IL-6 is a cytokine that modulates the biological activity of a wide range of cells, including cancer cells. IL-6 has a role in the host's immunological response as well as the development and differentiation of a variety of malignant tumors, according to the USA National Cancer Institute. It has been revealed that the IL-6R-JAK-STAT3 signaling pathway is involved in the promotion of cancer development and progression [43]. STAT proteins are a class of transcription factors that play an important part in the signaling pathways involving tyrosine kinases [44]. When STAT3 is activated continuously, it may enhance cell cycle progression, tumor invasion, tumor cell death, metastasis, tumor proliferation, and angiogenesis, among other things.

Host genetic variables, including inflammation-induced cytokines, are crucial in the etiology, development, and prognosis of cervical cancer, as well as other cancers. In a study of 215 cervical cancer patients, the level of serum CRP is closely related to tumor stage, lymphatic metastasis, and age, but not cell grade and tissue type. This suggests CRP as a valuable prognostic parameter for cervical cancer due to its close relationship with tumor-free survival and overall survival [45]. In a prospective study, serum CRP level increased within a few years before the diagnosis of ovarian cancer. In the group with high serum CRP levels (3 mg/L ≤ CRP < 10 mg/L), the risk of ovarian cancer increases about twice [46]. These results explain that elevated CRP levels are related to worse clinical outcomes, including DFS, PFS, and OS. A substantial connection was found between CRPs and OS in the subgroup analysis with a cut-off value of ≥5 mg/L for CRPs. It has been proven that as the level of CRP increases, the prognosis becomes poorer.

The article "C-Reactive Protein as a Prognostic Biomarker for Gynecologic Cancers: A Meta-Analysis" was retracted in 2023. Reasons: signs of a paper mill; suspected computer-generated content; unreliable results or conclusions; concerns about the data.

Therefore, we believe that CRP can be used to guide the personalized care of gynecological cancer and as a reference factor for postoperative recurrence risk assessment and adjuvant treatment.

It is worth noting some evident limitations of the current study. Patients with gynecologic malignancies had a wide range of characteristics, including cancer kind, stage, treatment plan, and follow-up month, all of which might have a significant influence on the aggregated findings. Second, the cut-off value for CRP was derived using previously published data, which may have shown some variability in the data. Third, this meta-analysis contained just 19 articles. For this reason, well-designed studies with high sample sizes should be done in the future to confirm our findings, as previously stated.

## 5. Conclusions

A high serum CRP level is associated with a poorer prognosis for gynecologic cancers. Serum CRP, an easily obtained indicator, may be widely used to help predict the prognosis of patients.

## Figures and Tables

**Figure 1:** Flowchart of study selection.

**Figure 2:** Forest plot of the association between CRP level and FIGO stage (a), OS (b), DFS (c), and PFS (d) in gynecologic cancers. FIGO, International Federation of Gynecology and Obstetrics; DFS, disease-free survival; OS, overall survival; PFS, progress-free survival.

**Figure 3:** Analysis of subgroups for the association between CRP and OS. (a) Subgroup analysis based on cancer type. (b) Subgroup analysis based on HR. (c) Subgroup analysis based on serum CRP concentration measured before or after surgery. (d) Subgroup analysis based on country (Eastern or Western). (e) Subgroup analysis based on age. (f) Subgroup analysis based on the cut-off value of CRP. CRP: C-reactive protein.

**Figure 4:** Publication bias and sensitivity analysis of the studies selected. (a) Analysis of sensitivity for independent studies according to the correlation between the CRP level and FIGO stage; (b) analysis of sensitivity for independent studies according to the correlation between the CRP level and OS; (c) analysis of sensitivity for independent studies according to the correlation between the CRP level and DFS; (d) analysis of sensitivity for independent studies according to the correlation between the CRP level and PFS.

The article "C-Reactive Protein as a Prognostic Biomarker for Gynecologic Cancers: A Meta-Analysis" was retracted in 2023. Reasons: signs of a paper mill; suspected computer-generated content; unreliable results or conclusions; concerns about the data.

**Table 1:** Main characteristics of studies included in this meta-analysis.

First author, publication year	Country	Recruitment period	Age (mean/median) yr	No. pts	Cancer type	Pathology	Stage	Survival analysis	Mean/median months of follow-up	NOS scores
Schmid et al. 2007 [36]	Austria	1995–2005	NM	403	EC	ADC	FIGO I-IV	OS,DFS	NM	6
Six et al. 2008 [33]	Austria	1995–2003	69.1	67	VC	SCC	FIGO I-IV	OS,DFS	NM	7
Hefler et al. 2008 [28]	Austria	NM	60.5	623	OC	Serous, mucinous, endometrioid, clear cell, and others	FIGO I-IV	OS	25.5	7
Stephan et al. 2011 [23]	Austria	2000–2009	49.2	178	CC	SCC and non-SCC	FIGO I-IV	OS,DFS	46	8
Dobrzycka et al. 2013 [27]	Poland	2003–2007	57.6	118	OC	Serous, mucinous, endometrioid, clear cell, and others	FIGO I-IV	OS,DFS	24.63	8
Nakamura et al. 2015 [21]	Japan	2005–2014	52.6	32	CC	SCC and non-SCC	NM	OS	NM	7
Zhang et al. 2015 [29]	China	2000–2012	50.6	190	OC	Serous, mucinous, endometrioid, clear cell, and others	FIGO I-IV	OS,PFS	43	8
Lu et al. 2015 [31]	China	2006–2010	55.28	107	OC	serous, mucinous, endometrioid, clear cell, and others	FIGO I-IV	OS	28.5	8
Li et al. 2015 [34]	China	2007–2009	53	282	EC	Endometrioid and others	FIGO I-IV	DSS	51.2	8
Xiao et al. 2015 [26]	China	2004–2011	52	238	CC	SCC, non-SCC	FIGO IB1-IVA	OS,PFS	42	8
Bodner–Adler et al. 2016[19]	Austria	2005–2015	51	46	CC	ADC	FIGO I-IV	OS	NM	7
Liu et al. 2017 [32]	China	2006–2012	53	200	OC	Serous, mucinous, endometrioid, clear cell, and others	FIGO I-IV	OS	NM	8
He et al. 2018 [25]	China	2007–2009	69	198	CC	SCC	FIGO I-IV	OS	NM	8
Wang et al. 2019 [24]	China	2012–2014	51.5	110	CC	SCC	FIGO I-II	OS,PFS	NM	8
Wang et al. 2020 [20]	China	2013–2015	59	150	CC	SCC	FIGO IB2,IIA2-IIB, III	OS	39	8
An et al. 2020 [22]	China	2010–2017	45.5	278	CC	SCC, non-SCC	FIGO IB-IIA	OS,RFS	NM	8
Terlikowska et al. 2020[35]	Poland	2006–2012	69	176	EC	ADC	FIGO I-IV	OS	NM	7
Komura et al. 2020[30]	Japan	2007–2016	NM	308	OC	Serous, mucinous, endometrioid, clear cell, others	FIGO I-IV	DSS	NM	6
Njoku et al. 2021 [37]	United Kingdom	2010–2015	66	358	EC	Endometrioid and others	FIGO I-IV	OS,RFS	40	8

Abbreviations: ADC: adenocarcinoma; CC: cervical cancer; DFS: disease-free survival; DSS: disease-specific survival; EC: endometrial cancer; FIGO: International Federation of Gynecology and Obstetrics; NM: not mentioned; OC: ovarian cancer; OS: overall survival; PFS: progress-free survival; RFS: recurrence-free survival; SCC: squamous cell carcinoma; VC: vulvar cancer.

**Table 2:** HRs and 95% CIs of patient survival or cancer progression in association with CRP in eligible studies.

First author, publication year	Cut-off value (mg/L)	PFS/DFS/RFS/DSS HR (95% CI)	OS HR (95% CI)
Schmid et al. 2007 [36]	5	1.2 (1.1–1.3)	1.1 (1.05–1.3)
Six et al. 2008 [33]	5	4.3 (0.9–13.7)	NM
Hefler et al. 2008 [28]	10	1.81 (1.81–2.74)	1.81 (1.81–2.74)
Stephan et al. 2011 [23]	5	1.2 (1.1–1.4)	1.4 (1.2–1.8)
Dobrzycka et al. 2013 [27]	11.19	0.84 (0.72–2.84)	1.87 (0.58–2.87)
Nakamura et al. 2015 [21]	7	NM	1.858 (0.644–5.357)
Zhang et al. 2015 [29]	10	1.49 (1.096–2.027)	1.435 (1.023–2.013)
Lu et al. 2015 [31]	8	NM	2.18 (1.3–3.67)
Li et al. 2015 [34]	8.2	7.24 (3.27–16.02)	NM
Xiao et al. 2015 [26]	10	1.88 (1.32–2.68)	1.95 (1.31–2.88)
Bodner–Adler et al. 2016 [19]	5	NM	1.238 (1.064–1.441)
Liu et al. 2017 [32]	10	NM	1.005 (1.001–1.009)
He et al. 2018 [25]	10	NM	3.03 (1.34–6.82)
Wang et al. 2019 [24]	3.135	1.423 (0.866–2.338)	2.081 (1.096–3.953)
Wang et al. 2020 [20]	5	NM	2.208 (1.265–3.251)
An et al. 2020 [22]	NM	1.32 (0.49–3.14)	1.25 (0.84–1.81)
Terlikowska et al. 2020 [35]	NM	NM	1.22 (1.01–1.43)
Komura et al. 2020 [30]	7.6	1.96 (1.1–3.57)	NM
Njoku et al. 2021 [37]	5.5	1.13 (0.58–2.20)	1.68 (1.00–2.81)

Abbreviations: DFS: disease-free survival; DSS: disease-specific survival; HR: HR (high vs. low); NM: not mentioned; OS: overall survival; PFS: progress-free survival; RFS: recurrence-free survival.

The article "C-Reactive Protein as a Prognostic Biomarker for Gynecologic Cancers: A Meta-Analysis" was retracted in 2023. Reasons: signs of a paper mill; suspected computer-generated content; unreliable results or conclusions; concerns about the data.

**Table 3:** Association between CRP level and clinicopathological characteristics in gynecological cancer patients.

Clinical parameters	Number of studies (number of patients)	OR (95% CI)	*p* value
Age	4 (725)	0.93 (0.69–1.25)	0.346
FIGO stage	4 (725)	0.43 (0.19–1.00)	0.001
Grade	3 (615)	0.74 (0.52–1.05)	0.685
Node	3 (618)	0.91 (0.65–1.28)	0.186

Abbreviations: CI: confidence interval; CRP: C-reactive protein; OR: odds ratio.

## Data Availability

The data that are included in this article are made available from the corresponding author upon request.
